The article "Long non-coding RNA NORAD exhaustion represses prostate cancer progression through inhibiting TRIP13 expression via competitively binding to miR-495-3p" was published in 2020. Journal: Cancer Cell Int.

# Long non-coding RNA NORAD exhaustion represses prostate cancer progression through inhibiting TRIP13 expression via competitively binding to miR-495-3p

**DOI:** 10.1186/s12935-020-01371-z

**Published:** 2020-07-18

**Authors:** Fengling Chen, Ling Liu, Shuya Wang

**Affiliations:** 1 Department of Urology, Huaihe Hospital, Henan University, Kaifeng, 475000 Henan China; 2 Department of Surgery, Huaihe Hospital, Henan University, No. 115, Ximen Street, Longting District, Kaifeng, 475000 Henan China

**Keywords:** Prostate cancer, NORAD, miR-495-3p, TRIP13

## Abstract

**Background:**

Prostate cancer (PCa) is a malignant heterogeneous tumor that threatens men’s health. Long non-coding RNA activated by DNA damage (NORAD) and microRNA-495-3p (miR-495-3p) have been revealed to be concerned with the tumorigenesis and progression of diverse cancers. Nevertheless, the regulatory mechanism between NORAD and miR-495-3p in PCa is unclear.

**Methods:**

The expression of NORAD, miR-495-3p, and thyroid hormone receptor interactor 13 (TRIP13) mRNA was detected with quantitative real-time polymerase chain reaction (qRT-PCR). The levels of Bcl-2, Bax, Cleaved-casp-3, TRIP13, cyclin D1, and PCNA were detected through western blot analysis. The proliferation, apoptosis, migration, and invasion of PCa cells were assessed through 3-(4, 5-dimethylthiazol-2-yl)-2, 5-diphenyltetrazolium bromide (MTT), flow cytometry, or transwell assays. The relationship between NORAD or TRIP13 and miR-495-3p was confirmed via dual-luciferase reporter, RIP, or RNA pull-down assays.

**Results:**

NORAD and TRIP13 were upregulated while miR-495-3p was downregulated in PCa tissues and cells. Both NORAD silencing and miR-495-3p upregulation accelerated cell apoptosis and curbed cell proliferation, migration, and invasion in PCa cells. Also, NORAD silencing repressed tumor growth in vivo. Notably, NORAD modulated TRIP13 expression by competitively binding to miR-495-3p. Furthermore, miR-495-3p repression reversed NORAD knockdown-mediated effects on the malignant behaviors of PCa cells. Moreover, TRIP13 enhancement overturned the effects of miR-495-3p overexpression on the proliferation, apoptosis, migration, and invasion of PCa cells.

**Conclusion:**

NORAD depletion inhibited PCa advancement via the miR-495-3p/ TRIP13 axis, which provided a potential tactic for PCa treatment.

## Highlights

1. NORAD and TRIP13 were upregulated and miR-495-3p was downregulated in PCa tissues and cells.
2. NORAD knockdown promoted cell apoptosis and suppressed cell proliferation, migration, and invasion in PCa cells.
3. MiR-495-3p overexpression induced apoptosis and repressed proliferation, migration, and invasion of PCa cells.
4. NORAD regulated TRIP13 expression via competitively binding to miR-495-3p in PCa cells.

## Background

Prostate cancer (PCa) is a complex heterogeneous tumor of male and ranks second among common malignancies in men worldwide [1]. Currently, most patients with PCa can be effectively treated by various treatments, such as radical resection and radiotherapy [2]. Unfortunately, approximately 25% of PCa patients relapse within 5 years [3]. Moreover, the recurrence, metastasis and castration-resistant progression of PCa are the leading causes of PCa death [4]. Hence, it is imperative to explore new PCa progress mechanism to develop effective PCa diagnosis and treatment.

Long non-coding RNAs (lncRNAs) are a class of critical members of the non-coding RNA (ncRNA) family that are more than 200 nucleotides in length and have no protein coding function [5, 6]. Increasing evidence has reported that lncRNAs exert a critical role in pathological and physiological processes, such as tumorigenesis and organ formation [6, 7]. LncRNA activated by DNA damage (NORAD) is an outstanding lncRNA, which plays a vital role in chromosomal stability and DNA protection [8]. The abnormal expression of NORAD was connected with the advancement of various cancers. For instance, increased NORAD expression was related to the poor prognosis of bladder cancer [9]. Also, NORAD could regulate the migration and proliferation of osteosarcoma cells [10]. And high NORAD expression was associated with tumor progression in colorectal cancer [11]. Also, NORAD depletion repressed epithelial ovarian cancer advancement [12]. Furthermore, NORAD was concerned with the tumorigenesis of PCa [13]. Nevertheless, the regulatory mechanism of NORAD in PCa progression has been not been well explained.

MicroRNAs (miRNAs) are a class of short ncRNAs (approximately 22 nucleotides), which participate in a range of biological processes, such as cell differentiation, movement, proliferation, and apoptosis [14]. In recent years, miRNAs are revealed to be abnormally expressed in tumors and have attracted widespread attention [15]. MicroRNA-495-3p (miR-495-3p) was showed to be downregulated in a series of tumors, such as colon cancer [16], melanoma [17], and osteosarcoma [18]. MiR-495-3p served as a suppressor in gastric carcinogenesis via modulating multiple epigenetic modifiers [19]. Also, the lncRNA UCA1/miR-495-3p/SATB1 axis was related to cell invasion and proliferation in gastric cancer [20]. However, whether miR-495-3p can be regulated by NORAD has not been reported.

Thyroid hormone receptor interactor 13 (TRIP13), a member of the AAA + protein family, plays a pivotal role in mitosis [21, 22]. TRIP13 was revealed to be amplified in a variety of human cancers, and was concerned with tumor progression [23]. For instance, TRIP13 could accelerate tumor growth in colorectal cancer [24]. Furthermore, reduced TRIP13 expression curbed tumor metastasis and growth in hepatocellular cancer [25]. Also, TRIP13 was revealed as a predictor for poor prognosis of PCa [26]. Nevertheless, it is unclear whether NORAD and miR-495-3p can regulate the expression of TRIP13 in PCa.

Hence, we evaluated the expression patterns of NORAD, miR-495-3p, and TRIP13 in PCa tissues and cells. Moreover, the roles of NORAD and miR-495-3p in PCa cells in vitro were further investigated. Furthermore, we also explored the mechanism of the NORAD/miR-495-3p/TRIP13 axis in PCa, which provided a possible strategy for the treatment of PCa.

## Materials and methods

### PCa specimen collection

The current research was permitted by the Ethical Committee of Huaihe Hospital, Henan University. All specimens (PCa tissues and adjoining healthy tissues) used in this research were collected from 30 patients with PCa who were diagnosed at Huaihe Hospital, Henan University hospital. PCa patients participating in this research did not receive any treatment before surgery. Moreover, all participants in this research signed informed consents prior to surgery. The clinicopathological characteristics of patients with PCa were shown in Table 1.

**Table 1:** The clinicopathological characteristics of 30 prostate cancer patients

Clinicopathologic parameters	Case
Age (years)	
≤ 60	12
> 60	18
Tumor size	
≤ 2.5 cm	20
> 2.5 cm	10
Pathological stage	
I–II	19
III	11
Lymph node metastasis	
No	9
Yes	21
Histological grade	
G1 + G2	16
G3	14

### Cell culture

PCa cell lines (DU145, 22Rv1, and LNCaP) and the normal human prostate epithelial cells RWPE-1 were procured from American Tissue Culture Collection (Manassas, VA, USA). The Roswell Park Memorial Institute (RPMI) 1640 medium from Life Technologies (Grand Island, NY, USA) supplemented with fetal bovine serum (10%, FBS, HyClone, Logan, UT, USA), streptomycin (100 μg/mL, Life Technologies) and penicillin (100 U/mL, Life Technologies) was utilized to culture the above cell lines. Moreover, all cells were kept in an incubator with 5% CO_2_ at 37℃.

### Quantitative real-time polymerase chain reaction (qRT-PCR)

Total RNA of PCa tissues and adjoining healthy tissues, as well as cells, were extracted through TRIzol reagent (Thermo Fisher Scientific, Waltham, MA, USA). Primer-Script one step RT-PCR kit (Takara, Dalian, China) or MiRNA Reverse Transcription kit (Thermo Fisher Scientific) was employed to synthesize the first-strand complementary DNA. The levels of NORAD, miR-495-3p, and TRIP13 were assessed via SYBR Premix DimerEraser Kit (Takara). The primer sequences used in the research were presented as below: NORAD: 5′-TGATAGGATACATCTTGGACATGGA-3′ (F) and 5′-AACCTAATGAACAAGTCCTGACATACA-3′ (R); miR-495-3p: 5′-ACACTCCAGCTGGGAAACAAACATGGTGCA-3′ (F) and 5′-TGGTGTCGTGGAGTCG-3′ (R); TRIP13: 5′-ACTGTTGCACTTCACATTTTCCA-3′ (F) and 5′-TCGAGGAGATGGGATTTGACT-3′ (R); glyceraldehyde-3-phosphate dehydrogenase (GAPDH): 5′-GACTCCACTCACGGCAAATTCA-3′ (F) and 5′-TCGCTCCTGGAAGATGGTGAT-3′ (R); U6 small nuclear RNA (snRNA): 5′-GCTCGCTTCGGCAGCACA-3′ (F) and 5′-GAGGTATTCGCACCAGAGGA-3′ (R). The expression levels of NORAD, miR-495-3p, and TRIP13 were calculated by the 2^−ΔΔCt^ method, and GAPDH or U6 snRNA was viewed as an internal control for NORAD, TRIP13, and miR-495-3p.

### Cell transfection

Small interference RNA (siRNA) targeting NORAD (si-NORAD) and negative control (si-NC) were procured from GenePharma (Shanghai, China). The pcDNA-NORAD vectors (pcDNA-NORAD) and pcDNA-TRIP13 vectors (pcDNA-TRIP13) were constructed using the pcDNA3.1 vector (Invitrogen, Carlsbad, CA, USA). MiR-495-3p mimic (miR-495-3p) and scrambled mimics control (miR-NC), as well as miR-495-3p inhibitor (anti-miR-495-3p) and matching control (anti-miR-NC), were obtained from GenePharma. Also, the cells were transfected with Lipofectamine 2000 reagent (Invitrogen). The sequences were displayed as the following: si-NC (5′-GCGCGATAGCGCGAATATA-3′), si-NORAD (5′- AATAGAATGAAGACCAACCGC-3′), miR-495-3p (5′-TTTGTTTGTACCACGTGAAGAA-3′), and anti-miR-495-3p (5′-UUCUUCACGUGGUACAAACAAA-3′).

### 3-(4, 5-dimethylthiazol-2-yl)-2, 5-diphenyltetrazolium bromide (MTT) assay

The proliferation capacity of transfected PCa cells was evaluated through MTT assay. Briefly, transfected PCa cells (2.5 × 10^3^/well) were seeded into 96-well plates (Corning Costar, Corning, NY, USA) and maintained in an incubator with 5% CO_2_ at 37℃ for 24, 48, or 72 h. Then, MTT (20 μL) (Sigma, Louis, Missouri, USA) was replenished to each well and kept for 4 h. Thereafter, the supernatant of each well was discarded and dimethyl sulfoxide (150 μL, Sigma) was used for the dissolution of the formazan crystals. In the end, the Microplate Absorbance Reader (Thermo Fisher Scientific) was executed for the assessment of the optical density value at 490 nm.

### Flow cytometry assay

The apoptotic rate of transfected PCa cells was evaluated via the Annexin V-fluorescein isothiocyanate (FITC)/propidium iodide (PI) apoptosis detection kit (Sigma). In short, transfected PCa cells were cultured for 48 h. After washing with PBS, the cells were resuspended in binding buffer. Afterward, the binding buffer with transfected PCa cells (1 × 10^6^/mL) was supplemented with Annexin V-FITC (10 μL) and PI (5 μL) and kept for 15 min in the dark. At last, the FACScan flow cytometry from BD Biosciences (San Jose, CA, USA) was employed to analyze the apoptotic rate of transfected PCa cells.

### Western blot analysis

Total protein of PCa tissues and adjoining healthy tissues, as well as cells, was extracted by radio-immunoprecipitation assay (RIPA) lysis buffer (Thermo Fisher Scientific). Afterward, extracted protein was separated via the sodium dodecyl sulphate-polyacrylamide gel electrophoresis (10%, SDS-PAGE). After that, the wet electrophoretic transfer method was executed to transfer the separated protein onto polyvinylidene difluoride (PVDF) membranes (Millipore, Bedford, MA, USA). Next, the PVDF membranes were washed and then blocked by Tris Buffered Saline Tween (TBST) buffer with 5% skim milk. Then, the PVDF membranes were incubated with primary antibodies: anti-TRIP13 (HPA005727, Sigma), anti-GAPDH (1:2500, ab9485, Abcam, Cambridge, MA, USA), anti-Bcl-2-associated X (Bax) (1:1000, ab32503, Abcam), anti-B cell lymphoma 2 (Bcl-2) (1:2000, ab182858, Abcam), anti-Cleaved-caspase-3 (Cleaved-casp-3) (1:500, ab32042, Abcam), anti-cyclin D1 (1:200, ab16663, Abcam), and anti-proliferation cell nuclear antigen (PCNA) (1:1000, ab92552). Subsequently, the membranes were washed and incubated with goat anti-rabbit IgG (1:2000, ab97051, Abcam). GAPDH was regarded as a loading control. Finally, the ImageJ software from the National Institutes of Health (Bethesda, MD, USA) was used to visualize the bands.

### Transwell assay

The transwell chamber (8 μm) from Corning Costar was applied to evaluate the migration and invasion capacities of transfected PCa cells. For the migration assay, RPMI 1640 medium (200 μL) embracing transfected PCa cells (1.5 × 10^5^) were added to the top chamber. Synchronously, RPMI 1640 medium (800 μL) supplemented with FBS (10%) was added to the lower chamber as a chemoattractant. After culturing for 24 h, a cotton swab was used to eliminate the cells on the upper surface of the member. Afterward, the migrated cells on the lower surface of the membrane were fixed via methanol (100%) and stained with crystal violet (0.25%, Sigma). The invasion assay was performed with a transwell chamber coated with matrigel matrix (BD Biosciences). Eventually, the migrated or invaded cells were counted using a light microscope (Olympus, Tokyo, Japan).

### Dual-luciferase reporter assay

The starBase v2.0 database was utilized for the prediction of the binding sites between miR-495-3p and NORAD or TRIP13. The pGL3-control vector (Promega, Madison, WI, USA) with the wild type NORAD sequence (NORAD WT) and mutant NORAD sequence (NORAD MUT) (within predicted miR-495-3p binding sites) were constructed to verify the binding sites between miR-495-3p and NORAD. Similarly, the wild type TRIP13 3′-Untranslated Regions (UTR) and mutant TRIP13 3′-UTR sequences (within predicted miR-495-3p binding sites) were synthesized and inserted into the pGL3-control vector to construct the luciferase reporters. Afterward, the miR-NC or miR-495-3p was co-transfected into PCa cells with luciferase reporter vectors for the execution of the dual-luciferase reporter assay, respectively. Finally, the luciferase activities of luciferase reporter vectors were determined through the dual-luciferase reporter assay kit (Promega).

### RNA immunoprecipitation (RIP) assay

The relationship between miR-495-3p and NORAD was verified via the Magna RIP™ RNA Binding Protein Immunoprecipitation Kit (Millipore). In short, 22Rv1 and LNCaP cells were lysed in RIP lysis buffer with protease inhibitor (Sigma) and RNase inhibitor (Thermo Fisher Scientific). Then, the lysates were incubated in RIP buffer containing magnetic beads, and the magnetic beads were conjugated with anti-AGO2 or anti-IgG antibodies (Millipore). Subsequently, the magnetic beads were incubated with proteinase K (Sigma) for the digestion of the protein. Afterward, total RNA was isolated via the TRIzol reagent (Thermo Fisher Scientific). The enrichment of miR-495-3p and NORAD was evaluated through qRT-PCR.

### RNA pull-down assay

The biotinylated (bio)-NC and bio-miR-495-3p were acquired from Sigma Aldrich. In short, 22Rv1 and LNCaP cells were transfected with bio-NC or bio-miR-495-3p, respectively. Then, the cells were lysed with lysis buffer. Next, the lysate was incubated with streptavidin-coupled magnetic beads for 2 h. Thereafter, the bound RNA was obtained via using Trizol reagent, and the level of TRIP13 was determined via qRT-PCR.

### Xenograft assay

The animal experiments were approved by the Ethics Committee of Huaihe Hospital, Henan University. 18 BALB/c nude mice (5-week-old) were obtained from Shanghai Experimental Animal Center (Shanghai, China) and housed in no specific pathogentic conditions with water and food. LNCaP (2 × 10^6^) cells transfected with sh-NC, lentivirus-mediated sh-NORAD, or lentivirus-mediated sh-NORAD + anti-miR-495-3p was subcutaneously injected into the dorsal side of mice (6 mice in each group). Tumor volume was measured once a week using a digital caliper. The tumor volume was calculated with the equation:

$${\text{Volume}} = ({\text{length}}\times {\text{width}}^{2}/2)$$

On day 35, the mice were killed through cervical dislocation under 5% isoflurane for subsequent analysis.

### Statistical analysis

SPSS 20.0 software (IBM, Armonk, NY, USA) and GraphPad Prism 5.0 (GraphPad, San Diego, CA, USA) were employed for the conduction of the statistical analysis. Student’s *t* test or one-way variance analysis (ANOVA) was applied to compare the differences between two or among more groups. Differences with *P* < 0.05 were statistically significant. Pearson’s correlation analysis was utilized to assess the correlation among NORAD, miR-495-3p, and TRIP13 in PCa tissues. The data for this study were derived from at least 3 independent experiments and were shown as mean ± standard deviation.

## Results

### NORAD was augmented while miR-495-3p was downregulated in PCa tissues and cells

To assess the role of NORAD in PCa, we employed the qRT-PCR for the assessment of the expression level of NORAD in 30 paired PCa tissues and adjoining healthy tissues. The data exhibited that an apparent elevation of NORAD was discovered in PCa tissues compared to that in adjoining healthy tissues (Fig. 1a). Compared to the RWPE-1 cells, NORAD expression was strikingly increased in PCa cell lines (DU145, 22Rv1 and LNCaP). Furthermore, NORAD expression was higher in 22Rv1 and LNCaP cells than that in DU145 cells (Fig. 1b). Subsequently, the expression pattern of miR-495-3p in PCa tissues and cell lines was explored. As presented in Fig. 1c, d, miR-495-3p expression was conspicuously decreased in PCa tissues and cell lines in contrast to adjoining healthy tissues and RWPE-1 cells. These results indicated that the abnormal expression of NORAD and miR-495-3p in PCa might be related to the progression of PCa.

**Fig. 1:** Expression levels of NORAD and miR-495-3p in PCa tissues and cells. **a** QRT-PCR was employed to analyze the expression level of NORAD in 30 paired PCa tissues and adjoining healthy tissues. **b** The level of NORAD in PCa cell lines and RWPE-1 cells was assessed with qRT-PCR. **c**, **d** The expression of miR-495-3p in PCa tissues, adjoining healthy tissues, PCa cell lines, and RWPE-1 cells was detected using qRT-PCR. The experiments were performed in triplicate. ***P < 0.001

### NORAD downregulation induced cell apoptosis and repressed cell proliferation, migration, and invasion in PCa cells

In view of the above results, we transfected the si-NC or si-NORAD into 22Rv1 and LNCaP cells to silence the expression of NORAD. Results of qRT-PCR exhibited that NORAD expression was dramatically reduced in 22Rv1 and LNCaP cells transfected with si-NORAD compared to the si-NC control (Fig. 2a). MTT assay displayed that decreased NORAD expression apparently restrained the proliferation ability of 22Rv1 and LNCaP cells (Fig. 2b, c). Flow cytometry assay was then carried out and the results indicated that NORAD silencing evidently facilitated the apoptosis of 22Rv1 and LNCaP cells (Fig. 2d). Western blot analysis suggested that NORAD inhibition dramatically elevated the levels of Bax and Cleaved-casp-3 and reduced the level of Bcl-2 in 22Rv1 and LNCaP cells (Fig. 2e–h). Also, transwell assay showed that the migration and invasion capacities of 22Rv1 and LNCaP cells were obviously inhibited by NORAD downregulation (Fig. 2i, j). Collectively, these results indicated that NORAD knockdown expedited apoptosis and repressed proliferation, migration, and invasion of PCa cells.

**Fig. 2:** Effects of NORAD downregulation on the proliferation, apoptosis, migration and invasion of PCa cells. **a **The expression of NORAD in 22Rv1 and LNCaP cells was evaluated by qRT-PCR. **a**–**j** 22Rv1 and LNCaP cells were transfected with si-NC or si-NORAD. **b**, **c** MTT assay was executed for the detection of the proliferation of 22Rv1 and LNCaP cells. **d** Flow cytometry assay was performed to assess the apoptosis of 22Rv1 and LNCaP cells. **e**–**h** Western blot analysis was conducted for the assessment of the levels of Bax, Bcl-2, and Cleaved-casp-3 in 22Rv1 and LNCaP cells. **i**, **j** Transwell assay was employed to evaluate the migration and invasion capacities of 22Rv1 and LNCaP cells. The experiments were performed in triplicate. ***P < 0.001

### Elevated miR-495-3p expression induced apoptosis and impeded proliferation, migration, and invasion of PCa cells

To evaluate the role of miR-495-3p in PCa, we employed the gain-of-function experiments to analyze the effects of miR-495-3p overexpression on proliferation, apoptosis, migration, and invasion of PCa cells. In comparison to the miR-NC control, miR-495-3p expression was strikingly reinforced in 22Rv1 and LNCaP cells after miR-495-3p transfection (Fig. 3a). MTT assay showed that the proliferation of 22Rv1 and LNCaP cells was drastically suppressed by miR-495-3p overexpression (Fig. 3b, c). Also, flow cytometry assay disclosed that miR-495-3p elevation notably accelerated the apoptosis of 22Rv1 and LNCaP cells (Fig. 3d). Transwell assay manifested that miR-495-3p upregulation inhibited cell migration and invasion in 22Rv1 and LNCaP cells (Fig. 3e, f). Besides, western blot analysis exhibited that enhanced miR-495-3p expression conspicuously upregulated the levels of Bax and Cleaved-casp-3 and downregulated the level of Bcl-2 in 22Rv1 and LNCaP cells (Fig. 3g, j). Taken together, the results suggested that miR-495-3p enehancement could trigger cell apoptosis and constrain cell proliferation, migration, and invasion in PCa cells.

**Fig. 3:** Effects of miR-495-3p mimic on the proliferation, apoptosis, migration, and invasion of PCa cells. **a** QRT-PCR was conducted for the evaluation of the expression of miR-495-3p in both 22Rv1 and LNCaP cells. **a**–**j** 22Rv1 and LNCaP cells were transfected with miR-NC or miR-495-3p. **b**, **c** The proliferation capacity of 22Rv1 and LNCaP cells was determined with MTT assay. **d** The apoptotic rate of 22Rv1 and LNCaP cells was assessed using flow cytometry assay. **e**, **f** The migration and invasion capacities of 22Rv1 and LNCaP cells were detected using transwell assay. **g**–**j** The levels of Bax, Cleaved-casp-3, and Bcl-2 in 22Rv1 and LNCaP cells were measured by western blot analysis. The experiments were performed in triplicate. ***P < 0.001

### NORAD served as a sponge for miR-495-3p in PCa cells

In consideration of the above results, we further explored whether NORAD acted as a sponge for miR-495-3p in PCa cells. We found that NORAD held the potential binding sites for miR-495-3p through the starBase v2.0 database. Dual-luciferase reporter assay manifested that miR-495-3p overexpression strikingly reduced the luciferase activity of luciferase reporters with NORAD WT in 22Rv1 and LNCaP cells, while the luciferase activity of luciferase reporters with NORAD MUT did not change (Fig. 4b, c). RIP assay exhibited that the enrichment of NORAD and miR-495-3p was higher in Ago2-harboring beads compared with the control IgG (Fig. 4d, e). RNA pull-down assay displayed that NORAD was pulled down by bio-miR-495-3p in comparison to the control bio-NC (Fig. 4f). We found that NORAD expression was negatively correlated with miR-495-3p in PCa tissues (Fig. 4g). And miR-495-3p expression was markedly elevated in NORAD-silenced 22Rv1 and LNCaP cells and was reduced in 22Rv1 and LNCaP cells after transfection with pcDNA-NORAD (Fig. 4h). Together, these data indicated that NORAD acted as a sponge for miR-495-3p in PCa cells.

**Fig. 4:** NORAD negatively regulated miR-495-3p expression in PCa cells. **a** The binding sites between NORAD and miR-495-3p were predicted with starBase v2.0 database. **b**, **c** The luciferase activities of luciferase reporter vectors of NORAD MUT and NORAD WT in 22Rv1 and LNCaP cells transfected with miR-495-3p or miR-NC were determined with dual-luciferase reporter assay. **d**, **e** RIP assay was performed to verify the relationship between miR-495-3p and NORAD. **f** RNA pull-down assay was employed to determine whether NORAD can be pull-down by miR-495-3p in both 22Rv1 and LNCaP cells. **g** Pearson’s correlation analysis method was employed to assess the correlation between NORAD and miR-495-3p in PCa tissues. **h** The expression of miR-495-3p in both 22Rv1 and LNCaP cells transfected with si-NORAD, si-NC, pcDNA-NORAD or pcDNA was detected by qRT-PCR. The experiments were performed in triplicate. ***P < 0.001

### MiR-495-3p inhibition weakened NORAD downregulation-mediated effects on proliferation, apoptosis, migration, and invasion of PCa cells

Given that NORAD negatively regulated the expression of miR-495-3p in PCa cells, we further explored whether NORAD played its function in PCa cells via miR-495-3p. The results presented that miR-495-3p expression was enhanced in NORAD-silenced 22Rv1 and LNCaP cells, while this trend was overturned after anti-miR-495-3p transfection (Fig. 5a). MTT assay manifested that the suppression of proliferation of 22Rv1 and LNCaP cells caused by NORAD inhibition was mitigated by miR-495-3p downregulation (Fig. 5b, c). Also, flow cytometry assay suggested that the promotive influence of NORAD inhibition on apoptosis of 22Rv1 and LNCaP cells was alleviated by miR-495-3p exhaustion (Fig. 5d). Moreover, transwell assay revealed that miR-495-3p knockdown strikingly counteracted the suppressive influence of NORAD reduction on migration and invasion of 22Rv1 and LNCaP cells (Fig. 5e, f). In addition, western blot analysis suggested miR-495-3p reduction could abate the effects of NORAD inhibition on the levels of Bax, Cleaved-casp-3, and Bcl-2 of 22Rv1 and LNCaP cells (Fig. 5g–j). In a word, these results indicated that NORAD mediated the malignant behaviors of PCa cells through miR-495-3p.

**Fig. 5:** Reduced miR-495-3p expression mitigated NORAD knockdown-mediated influence on cell proliferation, apoptosis, migration and invasion in PCa cells. **a** QRT-PCR was conducted for the evaluation of the expression of miR-495-3p in 22Rv1 and LNCaP cells. **a**–**j** 22Rv1 and LNCaP cells were transfected with si-NORAD, si-NC, si-NORAD + anti-miR-NC, or si-NORAD + anti-miR-495-3p. **b**, **c** The proliferation of 22Rv1 and LNCaP cells was analyzed with MTT assay. **d** Flow cytometry assay was executed for the assessment of the apoptosis of 22Rv1 and LNCaP cells. **e**, **f** Teanswell assay was carried out for the detection of cell migration and invasion in 22Rv1 and LNCaP cells. **g**–**j** The levels of Bax, Cleaved-casp-3, and Bcl-2 in 22Rv1 and LNCaP cells were assessed with western blot analysis. The experiments were performed in triplicate. *P < 0.05, **P < 0.01, and ***P < 0.001

### TRIP13 acted as a target for miR-495-3p in PCa cells

To deeply understand the molecular mechanism of PCa, we applied the starBase v2.0 database to predict the possible target of miR-495-3p. The results presented that TRIP13 might be a target for miR-495-3p (Fig. 6a). Results of dual-luciferase reporter assay exhibited that the co-transfection of the luciferase reporters with TRIP13 3′-UTR-WT and miR-495-3p markedly inhibited the luciferase activity in 22Rv1 and LNCaP cells. However, there was no apparent difference in the luciferase reporters with TRIP13 3′-UTR-MUT (Fig. 6b, c). RNA pull-down assay exhibited that TRIP13 mRNA was pulled down by bio-miR-495-3p in contrast to the control group (Fig. 6d). Also the levels of TRIP13 mRNA and protein were overtly increased in PCa tissues compared with adjoining healthy tissues (6E and 6F). Compared the RWPE-1 cells, the levels of TRIP13 mRNA and protein were conspicuously elevated in 22Rv1 and LNCaP cells (Fig. 6g, h). Furthermore, TRIP13 and miR-495-3p expression had a negative correlation in PCa tissues (Fig. 6i). In addition, we found that the protein level of TRIP13 were remarkably elevated in 22Rv1 and LNCaP cells transfected with anti-miR-495-3p, while the levels of TRIP13 protein were evidently reduced in 22Rv1 and LNCaP cells transfected with miR-495-3p (Fig. 6j). In short, miR-495-3p targeted TRIP13 in 22Rv1 and LNCaP cells.

**Fig. 6:** MiR-495-3p targeted TRIP13 in PCa cells. **a** The binding sites of miR-495-3p in the 3′-UTR of TRIP13 were predicted with starBase v2.0 database. **b**, **c** Dual-luciferase reporter assay was carried out to detect the luciferase activity of luciferase reporter vector of TRIP13 3′-UTR-MUT or TRIP13 3′-UTR-MUT in 22Rv1 and LNCaP cells transfected with and miR-495-3p or miR-NC. **d** RNA pull-down assay was executed to verify the relationship between miR-495-3p and TRIP13. **e**, **f** QRT-PCR or western blot analysis was conducted to assess the expression of TRIP13 mRNA and protein in PCa tissues and adjoining healthy tissues. **g**, **h** The expression levels of TRIP13 mRNA and protein in 22Rv1, LNCaP, and RWPE-1 cells were detected by qRT-PCR or western blot analysis. **i** Pearson’s correlation analysis method was used to analyze the correlation between TRIP13 and miR-495-3p in PCa tissues. **j** The expression of TRIP13 protein in 22Rv1 and LNCaP cells transfected with anti-miR-495-3p, anti-miR-NC, miR-NC, or miR-495-3p was detected by western blot analysis. The experiments were performed in triplicate. ***P < 0.001

### TRIP13 overexpression reversed miR-495-3p upregulation-mediated impacts on proliferation, apoptosis, migration, and invasion of PCa cells

Based on the above findings, we investigated whether miR-495-3p exerted its function through TRIP13. The data exhibited that TRIP13 protein levels were downregulated in miR-495-3p-increased 22Rv1 and LNCaP cells, while this effect was reversed after transfection with TRIP13 (Fig. 7a). We discovered that TRIP13 overexpression abrogated the suppression of proliferation of 22Rv1 and LNCaP cells induced by miR-495-3p overexpression (Fig. 7b, c). Moreover, flow cytometry assay demonstrated that the reintroduction of TRIP13 recovered the accelerative influence of miR-495-3p elevation on apoptosis of 22Rv1 and LNCaP cells (Fig. 7d). Transwell assay displayed that TRIP13 upregulation overturned the prohibitive effect of miR-495-3p upregulation on migration and invasion of 22Rv1 and LNCaP cells (Fig. 7e, f). In addition, western blot analysis displayed that TRIP13 reintroduction abolished the upregulation of Bax and Cleaved-casp-3 and the downregulation of Bcl-2 in miR-495-3p-increased 22Rv1 and LNCaP cells (Fig. 7g, j). These results indicated that miR-495-3p exerted its function through regulating TRIP13 expression in PCa cells.

**Fig. 7:** MiR-495-3p played its function via regulation of TRIP13 expression in PCa cells. **a** Protein level of TRIP13 in 22Rv1 and LNCaP cells was assessed using western blot analysis. **a**–**j** 22Rv1 and LNCaP cells were transfected with miR-NC, miR-495-3p, miR-495-3p + pcDNA or miR-495-3p + pcDNA-TRIP13. **b**, **c** MTT assay analysis of cell proliferation capacity in 22Rv1 and LNCaP cells. **d** Flow cytometry assay was applied to detect the apoptotic rate of 22Rv1 and LNCaP cells. **e**, **f** The migration and invasion abilities of 22Rv1 and LNCaP cells were evaluated with transwell assay. **g**–**j** The levels of Bax, Cleaved-casp-3 and Bcl-2 in 22Rv1 and LNCaP cells were analyzed through western blot analysis. The experiments were performed in triplicate. *P < 0.01 and ***P < 0.001

### NORAD regulated TRIP13 expression via targeting miR-495-3p in PCa cells

In light of all the above results, we next probed into whether NORAD could regulate TRIP13 expression as a competing endogenous RNA (ceRNA) in PCa cells. In the first place, we observed TRIP13 protein level was reduced in NORAD-decreased 22Rv1 and LNCaP cells, while this decrease was overturned by miR-495-3p silencing (Fig. 8a). Besides, TRIP13 could be pulled down by bio-NORAD (Fig. 8b). Also, the expression of NORAD and TRIP13 had a positive correlation in PCa tissues (Fig. 8c). Also, TRIP13 protein level was effectively downregulated in 22Rv1 and LNCaP cells after transfecttion with si-NORAD, while this reduction was overturned by TRIP13 reintroduction (Fig. 8d). And TRIP13 overexpression overturned the suppressive effect of NORAD downregulation on proliferation of 22Rv1 and LNCaP cells (Fig. 8e, f). Furthermore, the stimulative effect of NORAD knockdown on apoptosis of 22Rv1 and LNCaP cells was recovered by TRIP13 upregulation (Fig. 8g). In addition, TRIP13 elevation reversed the repression of migration and invasion of 22Rv1 and LNCaP cells caused by NORAD silencing (Fig. 8h, i). Also, elevated TRIP13 expression reversed the effects of NORAD inhibition on the levels of Bax, Cleaved-casp-3, and Bcl-2 of 22Rv1 and LNCaP cells (Fig. 8j–m). In sum, NORAD exerted its role by regulating TRIP13 expression via sponging miR-495-3p in PCa cells.

**Fig. 8:** NORAD bound to miR-495-3p to regulate TRIP13 expression. **a** The expression of TRIP13 protein in 22Rv1 and LNCaP cells transfected with si-NC, si-NORAD, si-NORAD + anti-miR-NC or si-NORAD + anti-miR-495-3p was evaluated with western blot analysis. **b** RNA pull-down assay was employed to verify the relationship between NORAD and TRIP13.  **c** Pearson’s correlation analysis revealed the correlation  between NORAD and TRIP13 expression in PCa tissues. **d** Western blot analysis was conducted to assess TRIP13 protein level in 22Rv1 and LNCaP cells. **d**-**m** 22Rv1 and LNCaP cells were transfected with si-NC, si-NORAD, si-NORAD + pcDNA or si-NORAD + pcDNA-TRIP13. **e**, **f** The proliferation of 22Rv1 and LNCaP cells was detected with MTT assay. **g** The apoptosis of 22Rv1 and LNCaP cells was analyzed via flow cytometry assay. **h**, **i** The migration and invasion capacities of 22Rv1 and LNCaP cells were assessed through transwell assay. **j–m** Western blot analysis was executed to evaluate the levels of Bax, Cleaved-casp-3 and Bcl-2 protein in 22Rv1 and LNCaP cells. The experiments were performed in triplicate. *P < 0.05, **P < 0.01, and ***P < 0.001

### NORAD depletion curbed tumor growth through the miR-495-3p/TRIP13 axis in vivo

Given that NORAD modulated TRIP13 expression through miR-495-3p in PCa cells in vitro, we further confirmed the regulatory mechanism in vivo through xenograft assay. We observed that NORAD expression was overtly decreased in LNCaP cells infected with lentivirus-mediated sh-NORAD compared to the sh-NC control, but this influence did not change after anti-miR-495-3p introduction (Fig. 9a). Moreover, miR-495-3p expression was elevated in LNCaP cells infected with lentivirus-mediated sh-NORAD compared to the lentivirus-mediated sh-NORAD + anti-miR-495-3p and sh-NC (Fig. 9b). Also, tumor volume and weight were decreased in mice tumor tissues of the sh-NORAD group, and this this repressed was partly recovered by the introduction of anti-miR-495-3p (Fig. 9c–e). And NORAD was downregulated in mice tumor tissues of the sh-NORAD group compared to the control group, and NORAD expression in mice tumor tissues of the sh-NORAD + anti-miR-495-3p group was consistent with the sh-NORAD group (Fig. 9f). Furthermore, the level of miR-495-3p was increased and the levels of TRIP13 mRNA and protein were reduced in mice tumor tissues of the sh-NORAD group, while this trend was partly abolished in mice tumor tissues of the sh-NORAD + anti-miR-495-3p group (Fig. 9g–i). Additionally, the levels of cyclinD1 and PCNA in mice tumor tissues of sh-NC, sh-NORAD, and sh-NORAD + anti-miR-495-3p groups were consistent with the TRIP13 mRNA and protein levels (Fig. 9j). Collectively, these results manifested that NORAD inhibition could constrain tumor growth in vivo through the miR-495-3p/TRIP13 axis.

**Fig. 9:** NORAD silencing repressed tumor growth through the miR-495-3p/TRIP13 axis in vivo. **a**, **b** The expression levels of NORAD and miR-495-3p in LNCaP cells transfected with sh-NC, sh-NORAD, or sh-NORAD + anti-miR-495-3p were detected with qRT-PCR. **c** Tumor volume was measured once a week in mice of the sh-NC, sh-NORAD, or sh-NORAD + anti-miR-495-3p groups. **d** A graph showing the tumor size of mice. **e** Tumor weight of mice of the sh-NC, sh-NORAD, or sh-NORAD + anti-miR-495-3p groups was assessed on day 35. **f**–**h** The expression of NORAD, miR-495-3p, and TRIP13 mRNA in tumor tissues of mice of the sh-NC, sh-NORAD, or sh-NORAD + anti-miR-495-3p groups was examined by qRT-PCR. **i**, **j** The levels of TRIP13 prtoein, cyclin D1, and PCNA in mice tumor tissues of the sh-NC, sh-NORAD, or sh-NORAD + anti-miR-495-3p groups were detected through western blot analysis. **P < 0.01 and ***P < 0.001

## Discussion

PCa has high morbidity and mortality. It was estimated that there will be 174,650 new cases of PCa and 31,620 deaths in the United States in 2019, and the number of new PCa cases and deaths will increases by 6 and 7% respectively over the previous year [27]. LncRNAs have been reported as therapeutic targets for some cancers, including PCa [28, 29]. Increased studies revealed that NORAD expression was elevated in various cancers. Li et al. revealed that NORAD expression was elevated in pancreatic cancer tissues, and NORAD silencing impeded metastasis and epithelial-to mesenchymal-transition (EMT) of pancreatic cancer cells in vivo and in vitro [30]. Another research revealed that NORAD was upregulated in colorectal cancer tissues, and NORAD inhibition induced apoptosis and constrained invasion, migration, and proliferation of colorectal cancer cells [31]. Zhang et al. stated that NORAD exhaustion constrained migration, proliferation, and accelerated apoptosis of PCa cells [13]. We also observed that NORAD expression was boosted in PCa tissues and cells. Furthermore, NORAD downregulation facilitated apoptosis and repressed proliferation, migration, and invasion of PCa cells. Our results were consistent with the above studies, revealing that NORAD played a carcinogenic role in PCa.

Increasing studies demonstrated that NORAD played its role in cancers via acting as a ceRNA [12, 32, 33]. MiR-495-3p was revealed to exert a suppressive role in a range of cancers. One report revealed that miR-495-3p upregulation could repress cell migration, invasion, and proliferation in osteosarcoma cells [18]. Wang et al. reported that lncRNA LUCAT1 depletion increased miR-495-3p expression in clear cell renal cell cancer cells, which could suppress cancer cell invasion and proliferation [34]. Li et al. discovered that increased miR-495 expression suppressed the invasion and migration of PCa cells via regulating mTOR and Akt signaling [35]. Consistent with the above studies, we observed that miR-495-3p was decreased in PCa tissues and cells. Also, miR-495-3p elevation promoted cell apoptosis and inhibited cell proliferation, migration, and invasion in PCa cells. NORAD acted as a sponge for miR-495-3p in PCa cells. Moreover, the proliferation, apoptosis, migration, and invasion of PCa cells mediated by NORAD downregulation were overturned by miR-495-3p silencing. Furthermore, NORAD inhibition reduced tumor growth in vivo, while this decrease was partly abolished by miR-495-3p inhibitor. Silenced NORAD expression decreased the levels of cyclinD1 and PCNA in mice tumor tissues, but this reduced overturned by miR-495-3p silencing. Mounting researches have revealed that cyclinD1 modulates G1 to S phase progression and is highly expressed in diverse tumors [36–38]. PCNA is a key medium in the process of DNA replication and can be used as a proliferation marker to evaluate the cell proliferation of xenograft tumor cells [39, 40].These data indicated that NORAD regulated cell malignant behaviors via sponging miR-495-3p in PCa.

It is well known that miRNA works by targeting its target genes. Previous researches reported that TRIP13 exerted a cancerogenic role in a series of cancer [41–43]. Report of Dong et al. claimed that TRIP13 was enhanced in PCa tissues and cells, and augmented TRIP13 expression accelerated invasion, migration, and proliferation of PCa cells [26]. Also, Zhang et al. revealed that miR-515-5p repressed the expression of TRIP13 in PCa cells, which repressed cancer cell invasion, migration, and proliferation [44]. Herein, TRIP13 was upregulated in PCa tissues and cells. Furthermore, TRIP13 depletion could expedite cell apoptosis and hamper cell proliferation, migration, and invasion in PCa cells. TRIP13 served as a target for miR-495-3p in PCa cells. TRIP13 overexpression weakened the effects of the miR-495-3p enhancement on cell proliferation, apoptosis, migration, and invasion in PCa cells. Therefore, we concluded that NORAD exhaustion decreased TRIP13 expression via sponging miR-495-3p in PCa cells, which repressed cell proliferation, migration, and invasion and accelerated cell apoptosis.

## Conclusion

All in all, NORAD depletion repressed PCa advancement via regulation of the miR-495-3p/TRIP13 axis. Furthermore, the research provided a might clue for the treatment of PCa.

## Data Availability

All data generated or analysed during this study are included in this published article.

## Abbreviations

PCa: Prostate cancer
miR-495-3p: MicroRNA-495-3p
TRIP13: Thyroid hormone receptor interactor 13
qRT-PCR: Quantitative real-time polymerase chain reaction
lncRNAs: Long non-coding RNAs
ncRNA: Non-coding RNA
